# Effects of ShenLing BaiZhu San Supplementation on Gut Microbiota and Oxidative Stress in Rats with Ulcerative Colitis

**DOI:** 10.1155/2021/3960989

**Published:** 2021-10-01

**Authors:** Daxing Gu, Shanshan Zhou, Lili Yao, Ying Tan, Xingzi Chi, Dayou Shi, Shining Guo, Cui Liu

**Affiliations:** ^1^College of Veterinary Medicine, South China Agricultural University, Guangzhou 510642, China; ^2^Guangdong Technology Research Center for Traditional Chinese Veterinary Medicine and Nature Medicine, Guangzhou 510642, China; ^3^International Institute of Traditional Chinese Veterinary Medicine, Guangzhou 510642, China

## Abstract

The aim of this study was to evaluate the effect of gut microbiota and antioxidation of Shenling Baizhu San (SLBZS) as a supplement in a rat model of ulcerative colitis (UC) induced by 2,4,6-trinitrobenzenesulfonic acid (TNBS). Acute intestinal inflammation was induced in 40 male SD rats aged 4 weeks with 100 mg/kg TNBS, and then three dosages of SLBZS (0.5 g/kg, 1 g/kg, and 1.5 g/kg) were administered for eight days, respectively. Faecal microbiome composition was assessed by 16S rRNA high-throughput sequencing. The result indicated that SLBZS could reduce the diversity of gut microbiota and increased its abundance. At the genus level, the relative abundance of SCFAs producing bacteria including *Prevotella* and *Oscillospira* increased, while the relative abundance of opportunistic pathogens including *Desulfovibrio* and *Bilophila* decreased. Meanwhile, SLBZS could improve the lesions of colon and significantly reduce the level of MPO, increase the levels of SOD and CAT in rats' serum. These findings revealed that SLBZS was effective and possessed anticolitic activities in a rat model of UC by reducing macroscopical and microscopical colon injury, enhancing antioxidant capacity, and regulating gut microbiota.

## 1. Introduction

UC, as a chronic, relapsing, and remitting inflammation of the gastrointestinal tract with high morbidity, brings a lot of pain to patients [1]. Gut microbiota was considered to be a critical factor in deriving UC [2, 3], which was characterized by abnormal microbiota leading to disruption of flora balance, decreasing the complexity of the intestinal microbial ecosystem [4]. At the same time, UC was thought to be caused by an imbalance between intestinal microbiota and mucosal immunity [5]. Among UC patients, the composition and functional diversity of intestinal microbiota and the stability of intestinal bacteria were reportedly destroyed [6]. Furthermore, the specific *Firmicutes* decreased, yet *Bacteroidetes* and *Lactobacillus* increased [7]. Hence, looking for supplements with a protective effect on gut microbiota needs to be urgently developed.

Studies have shown that some traditional Chinese medicine could modulate the composition of the gut microbiota and the gut microenvironment [8–10]. Meanwhile, the gut microbiota was essential for the metabolism of traditional Chinese medicine *in vivo* [11, 12]. SLZBS originated from the Song Dynasty “Taiping Huimin Mixing Agent,” composed of *Panax Ginseng*, *Poria cocos, Atractylodes macrocephala*, *Dioscorea opposita*, *Dolichos Lablab*, *Semen Nelumbinis*, *Semen Coicis*, *Fructus Amomi*, *Platycodon grandiflflorus*, and *Glycyrrhiza uralensis Fisch*. Modern pharmacological studies have revealed that many components of SLBZS contain anti-inflammatory activities. Ginseng polysaccharides, one of the constituents of *Panax Ginseng*, improved intestinal metabolism and absorption of ginsenosides [13]. Furthermore, Ginsenoside Rg1, also one of the main constituents of *Panax ginseng*, and its metabolites could inhibit colitis [14]. 16*α*-Hydroxytrametenolic acid from *Poria cocos* improved intestinal barrier function [15]. Yam polysaccharide from *Dioscorea opposita* reduced inflammation in the rat model of colitis induced by TNBS [16]. Polysaccharides from *Atractylodes macrocephala* could ameliorate ulcerative colitis via extensive modification of gut microbiota and host metabolism [17]. Moreover, it has been reported that SLBZS, by means of application of the combination, could treat UC in a significant way [18]. Besides, research shows that SLBZS could regulate the pathogenesis of UC with reduction of inflammatory cytokines, inhibition of pyroptosis, and protection of colonic barrier integrity [19, 20]. Currently, there was no uniform conclusion on the effect of UC on gut microbiota, and the traditional Chinese medicine SLBZS treats UC, which has not been theoretically explained. Recent studies have suggested that SLBZS, a complementary and alternative supplementary therapy for UC, could alleviate clinic symptoms by the improvement of biochemical criteria and restoration of intestinal barrier function [13]. SLBZS as a famous Chinese herbal formula has been reportedly used to treat UC, of which mechanism is unknown.

TNBS used to establish the UC model is a common modeling method [21]. In this study, TNBS was used to induce the UC model to evaluate the efficacy and safety of SLBZS in the treatment of UC, which provides a theoretical basis for the development of supplement during UC treatment. And then, fecal samples were collected on day 10 to identify the change of structure and diversity of the gut microbiota in response to the SLBZS treatment for the alleviation of UC. Furthermore, the levels of serum inflammatory factors and activity of antioxidant enzymes were measured, and the pathological changes of colon in UC rats were observed.

## 2. Materials and Methods

### 2.1. Preparation of TNBS and SLBZS

5% TNBS was purchased from Sigma-Aldrich Co., Ltd. 5% TNBS and 50% ethanol were mixed (1 : 1) when using. The traditional Chinese medicine prescription SLBZS, purchased from Beijing Tongrentang (Lot no: 16101034), comprises *Panax Ginseng*, *Poria cocos*, *Atractylodes macrocephala*, *Dioscorea opposita*, *Dolichos Lablab*, *Semen Nelumbinis*, *Semen Coicis*, *Fructus Amomi*, *Platycodon grandiflorus,* and *Glycyrrhiza uralensis Fisch*, and is dissolved in distilled water when used.

### 2.2. Experimental Animals

80 g∼100 g SD male rats aged 4 weeks were purchased from the Center of Experimental Animals of Southern Medical University (approval number: SCXK 2016-0041). All rats were housed in plastic cages with the ambient temperature controlled at 22°C∼24°C with light for 12 hours and free drinking water and food. The bottom of the cages lined with white paper made it easy to observe the stool. The padding was replaced every day during the test. All the experimental procedures of this study were approved by the Animal Ethics Committee of the South China Agricultural University (Guangzhou).

### 2.3. Experimental Design

After 5 days of adaptive feeding, 40 male rats were randomly divided into normal control group (CON), model group (TNBS), low dosage of SLBZS group (TNBS-L), medium dosage of SLBZS group (TNBS-M), and high dosage of SLBZS group (TNBS-H) (*n* = 8). All rats were weighed one day ahead of modeling and were fasted except water in 12 h before modeling. The CON group was treated with normal physiological saline, whereas all other rats were provided 100 mg/kg TNBS by transrectal for a single administration to induce acute UC. 2 days after modeling, rats in the CON group and TNBS group were intragastrically administered with physiological saline, and three dosages of SLBZS group were administered by oral gavage with SLBZS for 8 days, 0.5 g/kg SLBZS for rats in TNBS-L group, 1 g/kg SLBZS for rats in TNBS-M group, and 1.5 g/kg SLBZS for rats in TNBS-H group, respectively.

Then, feces were frozen immediately with liquid nitrogen and stored at −80°C. The abdominal aorta of anesthetized rats was dissected to collect blood samples, which were then separated for serum. Fresh colon tissues were collected in 10% formalin for investigation of histopathology.

### 2.4. High-Throughput 16S rRNA Gene Amplicon Sequencing

The total DNA of the feces was extracted using the TIANamp STool DNA Kit (Beijing, DP328). The extracted DNA was determined by 0.8% agarose gel electrophoresis, quantitatively analyzed by an ultraviolet spectrophotometer. Then, selected DNA was amplified by 16S rRNA V3-V4 region. The 16S rRNA V3-V4 region-specific primer for PCR amplification was 338F (5-barcode + ACTCCTACGGGAGGCAGCA-3'), 806R (5'-GGACTACHVGGGTWTCTAAT-3'). The PCR reaction system (25 *μ*L) was as follows: 0.25 *μ*L Q5 high-fidelity DNA polymerase PCR, 5 *μ*L reaction buffer (5×), 5 *μ*L high GC buffer (5×), 2 *μ*L NTP (10 mM), 2 *μ*L of template DNA, 1 *μ*L of each primer, 8.75 *μ*L of double distilled water. The PCR reaction conditions were 98°C for 30 s initially, followed by 25 cycles of denaturation at 98°C for 30 s, annealing at 50°C for 30 s and extension at 72°C for 30 s. The PCR amplification products were identified by electrophoresis, and then the amplified products were recovered and purified using the Axygen DNA Gel Recovery and Purification Kit. The products were sequenced on the Illumina MiSeq sequencing platform.

### 2.5. Bioinformatics and Statistical Analysis

QIIME was used for Operational Taxonomic Unit (OTU) classification and identification [22, 23]. Using R software to draw rarefaction curve, Alpha diversity index, including Chao1 estimator and Shannon diversity index are calculated. The principal component analysis (PCA) and weighted and unweighted nonmetric multidimensional scaling (NMDS) analysis based on UniFrac were carried out for community composition structure at genus level by R software [24, 25]. According to the statistics of the relative abundance of two levels of taxonomy, two levels of the phylum and the genus are analyzed.

### 2.6. Determination of Antioxidant Activity in Serum

Myeloperoxidase (MPO), superoxide dismutase (SOD), and catalase (CAT) levels of serum in each group were determined using ELISA kit according to the manufacturer's protocol (Shanghai Meilian Biological Technology Co., Ltd., Shanghai, China) (catalog numbers: ml003250, ml059387, and ml037079).

### 2.7. Histological Observation of Colon

The collected colon tissue was fixed in 10% formalin, dehydrated with different concentrations of ethanol, cleared with xylene, and embedded in paraffin. Paraffin-embedded tissues were cut into slices with a thickness of 5 *μ*m. For hematoxylin and eosin (HE) staining, paraffin‐embedded tissues were dewaxed, rehydrated, HE stained, dehydrated, cleared with xylene, and sealed. For TdT-mediated dUTP Nick-end Labeling (TUNEL) staining, slides were dewaxed, rehydrated, and incubated with proteinase K. Then, slides were washed with PBS to clear proteinase K. Following incubation with 3% H_2_O_2_ in PBS, slides were washed with PBS and then incubated with TUNEL reaction mix. The reactions were terminated by stop solution and then incubated with streptavidin HRP solution. After washing, slides were incubated with DAB chromogenic solution until a light brown background appeared. Following mounting, slides were observed under a light microscope.

### 2.8. Data Analysis

All data obtained in this study were processed statistically, and divergence was presented as means ± SE. One-way analysis of variance was used for multiple comparison with SPSS Statistics 20.0, and *P* < 0.05 was considered to be significantly different.

## 3. Results

### 3.1. Effect of the Structure of Intestinal Microbiota of Each Group after Treatment

After high-throughput sequencing, 1,707,839 effective sequences were obtained, including 307,951 in the CON group, 302,534 in the TNBS group, 383,561 in the TNBS-L group, 377,902 in the TNBS-M group, and 335,891 in the TNBS-H group. The QIIME software performed OTU partitioning on these sequences, which were based on 97% sequence similarity. Beta diversity analysis including PCA and weighted and unweighted NMDS based on UniFrac were used to analyze the similarity of the gut microbiota among different samples. PCA and NMDS analysis revealed that (Figures 1(a)–1(c)) the structure of gut microbiota in the TNBS group differed from the CON group. However, after administration of SLBZS, the structure of intestinal microbiota in the SLBZS group was similar to the CON group, particularly in the TNBS-M and TNBS-H group, which proved that administration of SLBZS could restore the intestinal structure of UC rats. The Chao1 and Shannon curves (Figures 1(d) and 1(e)) indicated that the curve tended to be flat when the sequencing depth was greater than 15000, proving that the sequencing depth was sufficient to reflect the species diversity and basically contained all species in the sample. The alpha diversity index (Figures 1(f) and 1(g)) showed that the Shannon diversity index in the TNBS-L group was lower than the CON group and TNBS group (*P* < 0.05), and Chao1 estimator in the SLBZS group was higher than that in the CON group and TNBS group (*P* > 0.05).

### 3.2. Taxonomic Composition of Communities at Phylum and Genus Levels after Treatment

The three typical microbiota at the phylum level were *Firmicutes*, *Bacteroidetes*, and *Proteobacteria* (Figure 2(a)). SLBZS treatment could increase the relative abundance of *Firmicutes* and *Proteobacteria* and reduce *Bacteroidetes* in UC rats (Figure 2(b)). At the genus level (Figure 2(c)), 6 of 110 genera were typically different after SLBZS treatment. In the TNBS-L and TNBS-H group, the relative abundance of *Prevotella* increased to normal level, but *Bilophila*, *Bacteroides*, and *Helicobacter* decreased compared to the TNBS group. In the TNBS-M group, the relative abundance of SLBZS *Oscillospira* was close to the normal level (Figure 2(d)).

### 3.3. Effect on Serum Antioxidant Enzymes after Treatment

As shown in Figure 3, SLBZS treatment could reduce the heightened activity of MPO induced by UC (*P* < 0.05). The SOD activity of TNBS-L and TNBS-M group was elevated compared to the TNBS group (*P* > 0.05). The CAT activity of the TNBS-L and TNBS-H group was elevated compared to the TNBS group (*P* > 0.05).

### 3.4. Histological Changes of Colon Tissue in Each Group after Treatment

Diarrhea, slightly rectal prolapse, and slightly colonic swelling were observed in TNBS-induced rats. After administration of SLBZS, the lesions of colon in UC rats were improved. The results illustrated that there was normal histological feature in the CON group, but a large number of infiltrated inflammatory cells and fuzzy structure of each layer in the TNBS group, and the structure of each layer of TNBS-H group was clearer and more integrated compared to the TNBS group, TNBS-L group, and TNBS-M group (Figure 4(a)). More apoptotic cells in the TNBS group compared to the SLBZS group were observed (Figure 4(b)). SLBZS reversed these changes.

## 4. Discussion

UC is a chronic inflammatory disease of colon with unclear mechanism. Generally, it has been believed that its pathogenesis involves the defect of epithelial barrier defects, dysregulated immune responses, and the disorder of intestinal microbiota. In TNBS-induced ulcerative colitis, UC rats are represented by diarrhea, ulceration of colon tissue, and enhancement of MPO activity in serum [26, 27]. In this study, all UC model rats demonstrated clinical symptoms of diarrhea. Concurrently, the disturbance of gut microbiota and antioxidant system existed in UC model rats, indicating the UC model was successfully established in this study.

Abnormal microbial composition and reduced complexity of the intestinal microbial ecosystem were common features of UC [28]. The present study showed that SLBZS supplementation could ameliorate dyspepsia and amend the dysregulated composition and function of the gut microbial community [29]. It contains different types of components with not only high nutritional value but also regulation of gut microbiota. To monitor the structural modulation of the gut microbiota during UC treatment with SLBZS, 16S rRNA high-throughput sequencing was performed in our study. As reflected by the Chao1 estimator study which also carried out a comparative analysis of the gimator and Shannon diversity index, we found that SLBZS treatment reduced the Shannon diversity index but increased the Chao1 estimator, suggesting SLBZS treated UC by reducing the diversity of gut microbiota while increasing its richness. PCA and NMDS showed that SLBZS treatment could change the structure and composition of the microbiota, and the structure of the microbiota can be closer to the normal state than the TNBS group. In order to analyze the further difference in the structure of gut microbiota after treatment, this study also carried out a comparative analysis of the gut microbiota at the phylum and genus levels of each group. We found that the relative abundance of *Bilophila*, *Desulfovibrio*, and *Bacteroides* decreased in TNBS-L and TNBS-H compared to the TNBS group, while *Oscillospira* and *Helicobacter* increased in TNBS-M, and *Prevotella* increased in the TNBS-L and TNBS-H group. *Prevotella* and *Oscillospira* were SCFA-producing bacteria [30, 31], and SCFA, important nutrients of colon mucosal, is capable of colon cell proliferation and mucosal growth [32]. Undigested dietary fiber, protein and peptides, can be fermented through gut microbiota in the cecum and colon, resulting in the generation of SCFA. SCFA could induce intestinal epithelial cells to secrete IL-18, antimicrobial peptide, and mucin and upregulate the expression of tight junction to regulate the integrity of intestinal barrier [33]. Meanwhile, SCFA could induce neutrophil migration and enhance phagocytosis [34]. *Bacteroides* was involved in metabolism and nutrient absorption *in vivo* [35], but promotes inflammation in inflammatory bowel disease [36]. Both *Desulfovibrio* and *Bilophila* were opportunistic pathogens, creating H_2_S in combination with H_2_ by sulfuric acid or sulfur-containing compounds, which has an important relationship with the inflammatory state of the intestinal epithelium (such as UC) [37]. Though *Helicobacter pylori* are defined as infectious pathogens according to Koch's law, studies have shown that *Helicobacter pylori* could regulate systematic immune homeostasis by inducing tolerogenic DCs and immunosuppressive Tregs. The body with *Helicobacter pylori* removed is more susceptible to colitis than the untreated group [38]. But infection of mice with *Helicobacter hepaticus* can cause colitis [39]. These suggest that the relationship between *Helicobacter* and IBD needs to be further revealed. Therefore, these results further indicated that the amelioration of UC using SLBZS may be mediated by the enrichment of bacteria to produce SCFA for the protection of colon mucosa and a reduction in bacteria, such as *Bacteroides*, *Desulfovibrio*, and *Bilophila*, to inhibit inflammation.

Colonic epithelial cells and mucosal barrier were strongly related to the pathogenesis of UC. By inhibiting the apoptosis of colonic epithelial cells, mucosal ulceration and mucosal epithelial cell damage in UC rats can be improved [1]. As a famous formula for 900 years, SLBZS has been widely used in the treatment of gastrointestinal diseases. It has been reported that SLBZS might exhibit ameliorating effects against diarrhea by modulations on intestinal absorption function as well as mucosal ultrastructure [40]. From the pathological section of the colon and the change of the colon in each group of the experiment, high dose of SLBZS for UC had a certain recovery effect on the intestinal villi detachment, the overall structural damage of the colon, inflammatory cell infiltration, and apoptosis induction, which was beneficial to regulate the reabsorption capacity and mucosal barrier of the colon. In addition, the activities of antioxidant enzymes in rats' serum were also ascertained. MPO was mainly located in aniline blue particles in neutrophils [41], which reflect the inflammatory state to some extent. Studies have found that reactive oxygen species (ROS) was closely related to UC colon mucosal tissue damage [42]. Although low level of ROS is necessary for some physiological processes, excessive ROS are produced in UC patients [43]. SOD and CAT can remove ROS, prevent lipid peroxidation, and maintain the stability of the cell membrane. In our study, we observed that low dosage of SLBZS treatment could decrease the level of MPO (*P* < 0.05) and increase the activities of SOD and CAT (*P* > 0.05). And, all dosage of SLBZS treatment could significantly decrease the level of MPO (*P* < 0.05) compared to the TNBS group. Our study proved that SLBZS could treat UC by enhancing antioxidant capacity, which may relate to recover the damaged colonic mucosa.

## 5. Conclusion

These findings revealed that SLBZS was effective and possess anticolitic activities as a supplement in a rat model of ulcerative colitis, by reducing macroscopical and microscopical colon injury, enhancing antioxidant capacity, and regulating gut microbiota. However, how SLBZS-mediated changes in the gut microbiota contribute to the improvement of UC needs further study.

## Figures and Tables

**Figure 1:** The effect on the intestinal microbiota structure of each group. (a) PCA analysis. (b) Unweighted NMDS analysis. (c) Weighted NMDS analysis. (d) Shannon curves. (e) Chao1 curves. (f) Shannon diversity index of each group. (g) Chao1 estimator of each group. ^a–c^Bars in the same index marked without the same letters differ significantly (*P* < 0.05).

**Figure 2:** Effect of taxonomic composition of communities in each group. (a) Histogram of microbial composition at the phylum level in each group. (b) Relative abundance of bacteria at the phylum level. (c) Histogram of microbial composition at the genus level in each group. (d) Relative abundance of bacteria at the genus level. ^a–c^Bars in the same index marked without the same letters differ significantly (*P* < 0.05).

**Figure 3:** Levels of serum antioxidant factors after treatment in each group. MPO, SOD, and CAT levels in UC rats. ^a-b^Bars in the same index marked without the same letters differ significantly (*P* < 0.05).

**Figure 4:** Histological changes of colon in each group. (a) HE staining (scale bar was 100 *μ*m). (b) TUNEL staining (scale bar was 100 *μ*m).

## Data Availability

We have deposited raw sequence data to support the findings of this study (e.g., in the NCBI Sequence Read Archive database) and added the information regarding data deposit. To see our data, use SRA RunSelector: http://www.ncbi.nlm.nih.gov/bioproject/752831. The numbers of Sequence Read Archive database are as follows. Submission ID: SUB10154324. BioProject ID: PRJNA752831.
